# Impact of Early Intravenous Haemostatic Drugs on Brain Haemorrhage Patients and Their Image Segmentation Based on RGB-D Images

**DOI:** 10.1155/2022/4608648

**Published:** 2022-01-07

**Authors:** Zhenzhen Wang, Yating Mou, Hao Li, Rui Yang, Yanxun Jia

**Affiliations:** Department of Neurology, Gucheng County Hospital, Hengshui 253800, China

## Abstract

Cerebral haemorrhage is a serious subtype of stroke, with most patients experiencing short-term haematoma enlargement leading to worsening neurological symptoms and death. The main hemostatic agents currently used for cerebral haemorrhage are antifibrinolytics and recombinant coagulation factor VIIa. However, there is no clinical evidence that patients with cerebral haemorrhage can benefit from hemostatic treatment. We provide an overview of the mechanisms of haematoma expansion in cerebral haemorrhage and the progress of research on commonly used hemostatic drugs. To improve the semantic segmentation accuracy of cerebral haemorrhage, a segmentation method based on RGB-D images is proposed. Firstly, the parallax map was obtained based on a semiglobal stereo matching algorithm and fused with RGB images to form a four-channel RGB-D image to build a sample library. Secondly, the networks were trained with 2 different learning rate adjustment strategies for 2 different structures of convolutional neural networks. Finally, the trained networks were tested and compared for analysis. The 146 head CT images from the Chinese intracranial haemorrhage image database were divided into a training set and a test set using the random number table method. The validation set was divided into four methods: manual segmentation, algorithmic segmentation, the exact Tada formula, and the traditional Tada formula to measure the haematoma volume. The manual segmentation was used as the “gold standard,” and the other three algorithms were tested for consistency. The results showed that the algorithmic segmentation had the lowest percentage error of 15.54 (8.41, 23.18) % compared to the Tada formula method.

## 1. Introduction

The disease burden of cerebral haemorrhage is not proportional to the proportion of stroke subtypes it accounts for. Although haemorrhagic stroke accounts for only 10%–15% and 20%–30% of all strokes in Europe, the USA, and Asia, respectively, it can cause death in approximately 40% of patients [1, 2]. There are more than 2 million strokes each year worldwide, with spontaneous cerebral haemorrhage accounting for about two-thirds of haemorrhagic strokes [3]. The incidence of cerebral haemorrhage, caused by small vessel disease in the brain, is thought to be related to the use of drugs, such as anticoagulants or antiplatelets, and increases with age, with approximately 2/3 of patients with cerebral haemorrhage over 75 years of age [4]. The prognosis for most of these patients is poor, with survival rates of 46% and 29% at 1 and 5 years after presentation. Old age, low Glasgow Coma Scale (GCS) score, a large haematoma size, ventricular haemorrhage, deep brain, and superficial haematoma are all risk factors for increased mortality [5]. Short-term haematoma enlargement occurs in approximately 26% of patients with cerebral haemorrhage [6], that is, an increase in haematoma volume of more than 33% of the basal haematoma volume or more than 6 ml [7], which is a major indicator of worsening neurological symptoms and death in the early stages of the disease [8]. Therefore, early hemostatic treatment of cerebral haemorrhage is essential to inhibit local fibrinolysis and activates coagulation mechanisms. Published clinical trials on hemostatic drugs for cerebral haemorrhage have not yielded conclusive evidence of clinical benefit, so in this article, we will discuss the mechanisms of haematoma expansion in spontaneous cerebral haemorrhage and the commonly used hemostatic drugs for clinical reference.

After a traumatic brain injury, the patients are all subject to abnormal stress responses in the early stages of the injury due to the severe mechanical forces to the head. Blood flow decreases as blood viscosity increases, platelet aggregation, and adhesion lead to increased local prothrombin concentrations, and the production of large amounts of fibrin promotes thrombus formation. Studies have shown that patients with traumatic brain injury have a high risk of coagulation abnormalities [9]. Patients with traumatic brain injury and cerebral haemorrhage are often in a state of stress, and changes in the internal environment affect cerebral blood flow and cerebral metabolic rate, which are often accompanied by a reduction in vascular self-regulation [10]. Studies have confirmed that abnormal blood flow severely affects microcirculatory perfusion, making the degree of ischaemia and hypoxia and organ damage more severe, and metabolic disorders follow, further aggravating the damage to the brain and neurological function. Therefore, for patients with cerebral haemorrhage from connoisseurs trauma, blood rheology is one of the most important indicators of the patient's disease status and is also a good indicator of the patient's treatment effect and prognosis.

Normal blood rheology in the body is a fundamental condition for the body to maintain normal haemodynamics for proper function and is an important factor in maintaining the homeostasis of the internal environment [11]. Abnormal blood rheology leads to microcirculatory abnormalities of blood rheology, causing the obstruction of microcirculation and hypoperfusion of tissues and organs and resulting in functional or organic disorders of the body, which in turn lead to metabolic disorders and aggravate brain damage [12]. Among the rheological indicators of blood, the concentration of macromolecular proteins contained in the plasma determines the viscosity of the plasma. Also, it influences the viscosity of whole blood at each shear rate. Also, the rate of oxygen transport in the blood is influenced by the viscosity of the blood [13]. An increase in the erythrocyte sedimentation rate, or hematocrit, often indicates the presence of vascular disease in patients. In this study, after treatment in both groups. A large number of experiments have pointed out that the blood rheology of patients with cerebral haemorrhage after connoisseur's trauma will undergo a series of changes, with the patients' blood viscosity and erythrocyte aggregation significantly increased. In contrast, the blood flow rate significantly decreased, resulting in blood stagnation and further aggravating the patients' cerebral ischaemia and hypoxia [8]. In this study, the better blood rheology index level in the observation group reflected the better microcirculatory status of the patients in the observation group after taking treatment. Therefore, the analysis of blood rheological indicators in patients with cerebral haemorrhage due to connoisseurs of trauma can directly reflect the blood circulation and inflammatory status of the body and help analyse the prognosis of the patient's condition.

In patients with acute connoisseurs trauma, most of whom are at risk of active bleeding, the choice of the therapeutic agent is very important. Edaravone is a free radical scavenger with potent hydroxyl radical scavenging and antioxidant effects and is commonly used clinically to alleviate the neurological symptoms associated with cerebral infarction and to protect damaged brain nerve cells, with a blood-brain barrier permeability of up to 60% [14]. Edaravone is widely used in clinical practice because it exists as an anion in the body, has a small molecular weight, can reduce the production of free radicals in multiple ways, and has a high blood-brain barrier permeability. Edaravone promotes the production of prostacyclin, inhibits xanthine oxidase, hypoxanthine oxidase, and leukorrhea production in vivo, removes highly cytotoxic hydroxyl groups, and shows the death of late neurons. All of these effects of earphone slow down the extent of damage to the blood-brain barrier. At the same time, earphone increases blood flow to brain tissue by slowing the stimulation of blood vessels by inflammatory factors and vascular stimulants [15].

## 2. Related Work

Rapid haemostasis after cerebral haemorrhage can prevent further expansion of the haematoma, which is beneficial in reducing the mortality rate and improving the neurological prognosis. The main treatments used in clinical practice include lowering blood pressure, correcting platelet and coagulation resistance (e.g., fisetin, prothrombin complex, platelets, fresh frozen plasma), and applying hemostatic drugs. Based on the principles of hemostatic drugs, it is appropriate to inhibit local fibrinolysis, activate coagulation, and not cause systemic thrombotic events. Antifibrinolytic agents include lysine, angiocarpic acid, traumatic acid, and synthetic derivatives of peptide-inhibiting peptidases, all of which inhibit fibrinolysis, stabilize the coagulation mechanism, and initiate haemostasis in the absence of cardiopathy [16], evaluating the efficacy and safety of angiocarpic acid in preventing early haematoma expansion after cerebral haemorrhage and concluding that it was safe for use in cerebral haemorrhage. Although the incidence of haematoma expansion within 12 hours of cerebral haemorrhage treated with angiocarpic acid did not differ significantly from the natural course of the disease, none of the cases included had serious adverse events such as cerebral, lower limb, or renal vein thrombosis, and there were no drug-related deaths. The effectiveness and safety of this drug in the treatment of spontaneous cerebral haemorrhage have yet to be demonstrated in a large randomised controlled clinical trial. The results of a group comparison of the effect of timing and dose of tragi-comic acid on the efficacy of treatment after CT diagnosis under strict control of blood pressure (target systolic blood pressure <150 mm Hg) showed that the incidence of haematoma enlargement was significantly lower in patients treated with antifibrinolytic drugs administered rapidly within 10 minutes of CT diagnosis (*p* < 0.05) and significantly more effective than in the group treated within 6 hours of CT diagnosis. However, the study included patients with cerebral haemorrhage who were all treated with the same regimen. There may be confounding factors that could affect the reliability of the results, so more randomised controlled trials are needed to validate the findings.

In addition, a recent meta-analysis showed that tragi-comic acid did not increase the risk of venous or arterial thrombosis [17]. In 2015, a small randomised controlled clinical trial from Malaysia used tragi-comic acid for the first time in patients with spontaneous cerebral haemorrhage and demonstrated that it was effective in preventing haematoma expansion [18]. A related clinical observation supports the conclusion that traumatic acid is effective in preventing haematoma enlargement in patients with spontaneous cerebral haemorrhage.

CT head examination can show the haemorrhagic foci well. However, the accurate estimation of the haematoma volume in CT images is a problem that needs to be solved in various studies. However, this method is time-consuming and laborious. With the advancement of AI technology, scholars have been attempting to automatically segment the haematoma volume in CT images. There are two main types of methods commonly used: fuzzy C-mean (FCM) clustering algorithms and neural networks. The FCM method is based on the grey-scale values of the CT images [19], improving the accuracy of the FCM segmentation method based on previous studies, but no large sample study has already validated its effectiveness. Neural network-based models have also been reported, to build an algorithm with 80% accuracy and 82% regression based on 30,000 head CT scans of brain haemorrhage images using a deep learning framework [20]. Most of the above studies were conducted from the perspective of artificial intelligence techniques. One computational method of [21], namely, segmentation of haematomas with the help of vocal random forest method, resulted in a consistency correlation coefficient (CCC) of 0.99 between this algorithm and manual segmentation in the validation set (30 cases), which was better than the Tada formula of 0.82. The difference between manual outlining, the Tada formula, and automatic segmentation did not reach statistical significance. In this study, based on the CT image characteristics of cerebral haematoma, we propose an algorithmic segmentation method based on deep learning technology-convolutional neural network (algorithmic segmentation) and compare it with the Tada formula and manual segmentation to initially explore the feasibility of an accurate and convenient cerebral haematoma segmentation method [22].

## 3. Semantic Segmentation of Cerebral Haemorrhage

### 3.1. RGB-D Sample Library Creation

In the representative brain haemorrhage dataset, firstly, representative stereo images of brain haemorrhage were selected from the dataset and the brain haemorrhage was divided into seven categories, which were not involved in the update calculation of weight during backpropagation [23]. The left RGB image in the stereo visual image was used as a sample, and each pixel of the image was labeled with the category to which it belonged, which was used as the label for training. Finally, the left RGB image and the parallax image D are fused into a four-channel RGB-D image. The final sample library consists of a training set, a validation set and a test set.

### 3.2. Network Training

In this paper, we implement semantic segmentation of RGB-D images of brain haemorrhage based on SegNet [24] and SegNet-Basic [25] networks. SegNet-Basic contains 8 convolutional layers, 4 downsampling layers, and 4 upsampling layers. Both network architectures are capable of end-to-end training and compared to other network architectures [26]. SegNet and SegNet-Basic can achieve higher semantic segmentation accuracy for semantic segmentation of brain haemorrhage and better real-time performance for semantic segmentation testing using the trained models.

The network is trained using a small batch training method, where a certain number of sample images are selected each time and fed into the network for forward propagation to obtain all the pixel points on the small batch sample images is calculated as the output error of the network [27].A cross-entropy loss function is used to calculate the training error of the network, which is calculated as

(1) $$\begin{array}{c} P\left(x=k\right)=\frac{\exp\left(a_{k}\right)}{\sum_{i}\exp\left(a_{i}\right)},\;i=0,1,\ldots ,K-1,\\ L=-\frac{1}{N}\sum_{i}\ln\left[P\left(x=k\right)\right],\;i=0,1,\ldots ,N-1. \end{array}$$

*P*(*x*=*k*) is the probability that pixel *x* belongs to its category *k*, *a*_*i*_ is the feature value of the *i*th category, obtained from the last convolutional layer, *K* is the number of categories classified, *N* is the number of all pixel points on a batch, and *L* is the training error value of the final output of the network. As the number of pixels occupied by each category on the training set varies widely, for example, the number of pixels occupied by pixel points such as sky and road is high, the median frequency balance [28] method is used to calculate the actual error values for different categories, calculated as

(2) $$\begin{array}{c} \lambda_{i}=\frac{m}{n_{i}},\;i=1,2,\ldots ,K. \end{array}$$

*λ*_*i*_ is the error value weight of the *i*th category, *n*_*i*_ is the number of pixels occupied by the *i*th category on the training set, and *m* is the median of the number of pixels occupied by each category. The optimised training error is calculated as

(3) $$\begin{array}{c} L=-\frac{1}{N}\sum_{i}\lambda_{i}\ln\left[P\left(x=k\right)\right],\;i=0,1,\ldots ,N-1. \end{array}$$

In the backpropagation phase of updating the network weight parameters, stochastic gradient descent is used to update the weight parameters of the network, which updates the weights by a linear combination of the negative gradient ∇*L*(*W*) and the last weight update value, calculated as

(4) $$\begin{array}{c} V_{t+1}=\mu V_{t}-\alpha \nabla L\left(W_{t}\right),\\ W_{t+1}=W_{t}+V_{t+1}. \end{array}$$

*W*_*t*_ is the weight matrix at the *t*th iteration, *V*_*t*_ is the weight update at the *t*th iteration, *α* is the base learning rate of the negative gradient, and *µ* is the weight of the weight update *V*_*t*_, which is used to weight the influence of the previous gradient direction on the current gradient descent direction [29]. Usually, during the iterative calculation, the base learning rate needs to be adjusted, the common adjustment strategies are fixed. When using the fixed method, the base learning rate remains unchanged during the iterative calculation. When using the step method, the relationship between the actual base learning rate *β* and *α* is

(5) $$\begin{array}{c} \beta =\alpha g^{\text{floor }}\left[\frac{a}{b}\right], \end{array}$$

where *a* is the number of current iterations, *b* is the step size of the base learning rate update, *g* is the base learning rate scaling factor, and *floor* is the upper rounding function. In order to reduce the probability of the network falling into local minima during training and verify the scalability and robustness of the algorithm, this paper uses two methods to train the network, fixed and step, setting *α* to 0.01 and *µ* to 0.9. When using the step learning strategy, *b* is set to 2 000 and *g* is set to 0.1; that is, for every 2 000 iterations, the basic learning rate is updated to the last 0.1 time.

## 4. Case Studies

### 4.1. General Information

Eighty patients with cerebral haemorrhage from cranial trauma treated in our hospital from November 2015 to February 2017 were equally divided into two groups by the random number table method: 40 patients in the observation group and 40 patients in the control group. In the observation group, there were 24 males and 16 females: age, (61.12 ± 3.28) years; duration of illness, (5.11 ± 2.16) years; BMI, (26.31 ± 7.27) kg/m^2^; site of haemorrhage, cerebellum in 4 cases, basal ganglia in 21 cases, thalamus in 7 cases, lobes in 8 cases; and mean volume of haemorrhage, (19.17 ± 8.73) mL [30]. In the control group, there were 23 males and 17 females: age, (60.86 ± 3.92) years; duration of disease, (5.05 ± 2.38) years; BMI, (26.28 ± 7.19) kg/m^2^; bleeding cerebellum in 5 cases; basal ganglia in 22 cases; thalamus in 6 cases; lobes in 7 cases; and average bleeding volume (18.86 ± 9.02) mL [31–33]. Exclusion criteria: (i) previous history of cerebral haemorrhage, stroke, cerebral infarction, and related haematological disorders; (ii) allergy to earphone; (iii) transient ischaemic attack and intracranial haemorrhage; (iv) primary cardiovascular, hepatic, renal, and haematopoietic disorders or severe mental disorders [34–36].

### 4.2. Results

The total clinical efficiency of the patients in the observation group was 95.00%, significantly higher than that of the control group, which was 72.50%, and the difference was statistically significant (*p* < 0.05) [37–39].  Table 1 shows a comparison of treatment results between the two groups.

After treatment, the FMA score (41.02 ± 10.12) and ADL score (53.86 ± 7.21) of the observation group were significantly higher than those of the control group, (33.72 ± 11.26) and (46.11 ± 7.92), with statistically significant differences (*p* < 0.05).  Table 2 presents a comparison of FMA and ADL scores between the two groups before and after treatment.

### 4.3. Comparison of Blood Rheology between Two Groups of Patients

After treatment, the whole blood viscosity (high cut and low cut), plasma viscosity sedimentation, platelet adhesion rate, and erythrocyte aggregation index of the observation group were significantly lower than those of the control group, and the difference was statistically significant (*p* < 0.05).  Table 3 displays a comparison of blood viscosity between the two groups before and after treatment.

After treatment, the NO level was significantly higher than that in the control group, as shown in Table 4. Table 4 is a comparison of changes in plasma ET and NO levels before and after treatment in the two groups.

## 5. Results

### 5.1. Data

The imaging data used in this study were obtained from the Chinese Intracranial Hemorrhage Imaging Database (CICHID). As of October 2019, nearly 5,000 head CT scans were collected from 22 medical centres (including 19 tertiary hospitals), including various types of intracranial haemorrhage such as cerebral parenchymal haemorrhage, ventricular haemorrhage, subdural haemorrhage, epidural haemorrhage, subarachnoid haemorrhage, and connoisseurs trauma, among which spontaneous cerebral parenchymal haemorrhage was the main type. In this study, some data on spontaneous parenchymal haemorrhage were selected for analysis.

The results of the consistency tests of the different methods are shown in Table 5 and Figure 1. Among the differences between the various methods and the manually segmented haematoma volume, the algorithmic segmentation had the narrowest range of differences at 17.90 ml; the exact Tada formula and the traditional Tada formula had a wider range of differences at 32.45 and 34.52 ml, respectively; the intragroup correlation coefficients between the three methods and the manual segmentation were all high (>0.75), but the intragroup correlation coefficients of 0.983 for the algorithmic segmentation and manual segmentation were higher than those of the two Tada formulae for manual segmentation (0.923 and 0.917).

In the light of the results of the above consistency tests, it can be concluded that the algorithmic split, the exact Tada formula, and the traditional Tada formula all have good consistency with the manual split, with the algorithmic split having a smaller fluctuation range than the two Tada formulae, while the exact Tada formula is slightly smaller than the traditional Tada formula.

In order to further analyse the reasons for the differences between the different methods of consistency testing, the study also explored whether the percentage errors of the different methods differed in different haematoma patterns (regular, irregular) and volumes (≥6 ml, <6 ml). In the validation set, 30 patients with spontaneous cerebral haemorrhage showed 18 regular and 12 irregular head CT images and 19 haematoma volumes ≥6 ml and 11 haematoma volumes <6 ml. As shown in Table 6, the percentage error of the exact Dota formula between the regular and irregular haematoma groups was statistically significant (*p*=0.038), suggesting that the percentage error of the formula differed among different haematoma morphologies. In contrast, the percentage error of the other methods differed between groups for different haematoma morphologies (regular versus irregular) or haematoma volumes (≥6 ml versus <6 ml).

The Tada formula is a simplification of the ellipsoidal volume formula (4/3 × *π* × 0.50 length × 0.50 width × 0.50 height), which is widely used for estimating cerebral haematoma volume because it is simple and quick to calculate. However, it tends to overestimate the volume of haematoma [26]. Previous studies suggested that the Tada formula cannot accurately estimate haematoma volume when the haematoma pattern is irregular or scattered [27]. This study showed that the percentage error seen in the calculation of the exact Tada formula was statistically different between regular and irregular haematomas. In contrast, the difference in the percentage error between the two types of the conventional Tada formula was not statistically significant. This may be related to the fact that the percentage error of the exact Tada formula is slightly smaller than that of the traditional Tada formula [17.49 (11.24, 43.01)% vs. 22.70 (14.53, 38.92)%]; that is, the percentage error of the traditional Tada formula is larger for both regular and irregular haematoma morphology. It was shown that the larger the haematoma volume (>40 ml versus 20∼40 ml), the larger the absolute and percentage error of the Tada formula [24]. The results of this study suggest that the percentage error of the Tada formula for estimating haematoma volume varies somewhat between haematoma forms but not between haematoma volume calculations, in line with the findings of [23]. It is worth noting that previous studies on computer-aided calculations comparing the Tada formula for estimating haematoma volume did not specify whether their studies used the Tada formula for estimation based on accurate computer measurements or the traditional film estimation method [24]. In contrast, the present study suggests that, compared with the traditional Tada formula for direct film estimation, the precise measurement of A, B, and C values with the help of tools in various medical imaging workstations has a smaller percentage error, a higher intragroup correlation coefficient, a narrower 95% LoA, and a higher agreement with manual segmentation results, allowing for a more accurate estimation of haematoma volume.

In order to obtain cerebral haemorrhage more accurately and quickly and compensate for the shortcomings of traditional computational methods, various algorithms for automatic haematoma segmentation were introduced, such as grey-scale clustering [17], Bayesian method [19], and random forest [25]. As the accuracy of different methods is shown in Figure 2, it can be known that depth learning algorithms are used for haematoma segmentation [17] with an accuracy of up to 80% [20]. However, computer engineering metrics such as accuracy and Dice values do not provide good answers to clinical questions such as measurement stability and comparative advantage over traditional methods. In this study, we explored the consistency of convolutional neural networks with manual segmentation and not only confirmed the accuracy of the former by the Bland–Altman consistency test and 95% LoA but also further validated the stability of the algorithm for different morphology and volumes of cerebral haematomas by a comparative analysis of haematoma morphology and volume sizes. Moreover, the convolutional neural network outperformed the conventional calculation method for cerebral haematoma volume compared to the Tada formula method.

The segmentation efficiency of different deep learning is shown in Figure 3. It is known that different deep learning amplification can be accurately and consistently calculate cerebral haematoma volume, which helps clinicians to better grasp the condition and answer clinical questions more precisely. In studies of the efficacy of surgery for cerebral haemorrhage, for example, there are sometimes contradictory conclusions in high-quality evidence. Although systematic evaluations, including Cochrane systematic reviews, concluded that surgery reduces morbidity and mortality, the large error in the traditional method of calculating haematoma volume (the Tada formula) may presumably be the reason for the contradiction between the high-quality evidence mentioned above. In addition to the accurate calculation of cerebral haematoma volume, the gradual implementation of automatic, accurate, and convenient cerebral haematoma segmentation with the intensive application of artificial intelligence technology in clinical medicine is the basis for further research in future computational methods such as imaging histology, surgical simulation, and surgical navigation.

As the research on convolutional neural network-based algorithm segmentation is still in its initial stage, it has certain limitations: (1) although the training set and validation set samples come from multicolor imaging data, the number is small, and the generalisation and generalisation ability of its algorithm still need further validation. (2) The number of cases was small, the haematomas in the validation set were skewed, nonparametric tests were used to compare the differences in haematoma volume and morphology, and the results need to be validated by expanding the sample size and using further tests of variability in future studies. (3) The small size of the haematoma in the validation set, averaging only 16 ml, led to a small absolute difference and an increase in the percentage error, resulting in an overestimation of the percentage error.

## 6. Conclusions

A segmentation method based on RGB-D images is proposed. Firstly, the parallax map D was obtained based on fused with RGB images to form a four-channel RGB-D image in order to build up a sample library. Secondly, the network was trained with 2 different learning rate adjustment strategies for 2 different structures of convolutional neural networks, respectively. Compared with the traditional Tada formula method, the convolutional neural network can calculate the volume of cerebral haematoma in head CT scan images with higher consistency and narrower 95% LoA than manual segmentation. Its percentage error varies less with different haematoma morphologies and volumes, which is promising for application, but still needs to be validated by a large sample clinical study.

## Figures and Tables

**Figure 1:** Bland–Altman consistency testing 1a. The algorithm segmentation has the narrowest 95% LoA of − 6.46∼5.97 ml, with 6.67% (2/30) of the points outside the 95% LoA.

**Figure 2:** Accuracy of different methods.

**Figure 3:** Segmentation efficiency of different deep learning.

**Table 1:** Comparison of treatment results between the two groups *n* (%).

Group	Remarkable effect	Effective	Invalid	Total effective rate
Observation group	23 (57.50)	15 (37.50)	2 (5.00)	38 (95.00)
Control group	12 (30.00)	17 (42.50)	11 (27.50)	29 (72.50)
*u*(*x*^2^)	2.9831		7.4397	
*p*	0.0029		0.0064	

**Table 2:** Comparison of FMA and ADL scores between the two groups before and after treatment ($\bar{x}\pm s$).

Group	FMA		ADL	
	Before treatment	After treatment	Before treatment	After treatment
Observation group	20.34 ± 11.79	41.02 ± 10.12	36.78 ± 6.12	53.86 ± 7.21
Control group	20.41 ± 12.82	33.72 ± 11.26	37.02 ± 5.98	46.11 ± 7.92
*T*	0.0254	3.0496	0.1774	4.5765
*p*	0.9798	0.0031	0.8597	0.0000

**Table 3:** Comparison of blood viscosity between the two groups before and after treatment ($\bar{x}\pm s$).

Group	Whole blood viscosity (high shear)		Whole blood viscosity (low shear)		Plasma viscosity (MPa/s)		ESR (mm/h)		Platelet adhesion rate (%)		Erythrocyte aggregation index	
	Before treatment	After treatment	Before treatment	After treatment	Before treatment	After treatment	Before treatment	After treatment	Before treatment	After treatment	Before treatment	After treatment
Observation group	4.49 ± 1.69	3.12 ± 0.53	9.12 ± 1.83	7.69 ± 1.57	1.61 ± 0.24	0.21 ± 0.15	25.28 ± 5.58	18.15 ± 4.24	43.28 ± 6.18	38.65 ± 6.24	7.66 ± 1.63	5.29 ± 1.178
Control group	4.68 ± 1.53	3.74 ± 0.76	9.08 ± 1.88	8.57 ± 1.38	1.59 ± 0.21	13.6 ± 0.37	25.23 ± 5.52	21.81 ± 6.21	43.23 ± 6.21	41.81 ± 6.21	7.88 ± 4.12	7.27 ± 1.08
*T*	0.5271	4.2321	0.0964	2.6626	0.3966	2.3762	0.0403	3.0789	0.0352	2.2702	0.6320	2.547
*p*	0.5996	0.0001	0.9234	0.0094	0.6927	0.0199	0.9680	0.0029	09720	0.0260	0.5292	0.0000

**Table 4:** Comparison of changes in plasma ET and NO levels before and after treatment in the two groups ($\bar{x}\pm s$).

Group	NO (pg/ML)		ET (moL/L)	
	Before treatment	After treatment	Before treatment	After treatment
Observation group	56.91 ± 11.82	78.12 ± 12.73	92.46 ± 15.53	72.19 ± 10.47
Control group	57.08 ± 12.13	70.56 ± 11.51	91.79 ± 15.48	82.87 ± 11.48
*T*	0.0635	2.7860	0.1932	4.3473
*p*	0.9495	0.0067	0.8473	0.0000

**Table 5:** Consistency tests for different measurement methods (*n* = 30, ml).

Haematoma difference	Algorithm for manual segmentation	Application of exact multifield formula to manual segmentation	Traditional multifield formula for manual segmentation
Range	−11.11–6.79	−8.39–24.06	−4.69–26.83
Average	−0.21	1.98	2.37
Median	0.15	−0.07	−0.15
95% LoA	−6.46–5.97	−12.55–16.51	−13.34–18.07
ICC (95%CI)	0.983	0.923	0.917

**Table 6:** Analysis of variability of different measurement methods in different haematoma morphologies and volumes [M (P25, P75), %].

Measuring method	Haematoma morphology		*Z* value	*p* value	Haematoma volume		*Z* value	*p* value
	Rule (*n* = 18)	Irregular (*n* = 12)			≥6 m (*n* = 19)	<6 m (*n* = 11)		
Algorithm segmentation	15.73	13.33	−0.085	0.933	14.31	21.04	1.442	0.149
Exact multifield formula	13.87	34.82	0.074	0.038	23.52	14.59	−0.882	0.378
Traditional multifield formula	21.87	26.17	0.085	0.933	22.70	21.52	1.140	0.254

## Data Availability

The simulation experiment data used to support the findings of this study are available from the corresponding author upon request.
